The article "Hippocampal neuronal cells that accumulate α-synuclein fragments are more vulnerable to Aβ oligomer toxicity via mGluR5 – implications for dementia with Lewy bodies" was retracted in 2025. Reasons: duplicated images; overlap with earlier publications; unreliable data; concerns about the data.

# Hippocampal neuronal cells that accumulate α-synuclein fragments are more vulnerable to Aβ oligomer toxicity via mGluR5 – implications for dementia with Lewy bodies

**DOI:** 10.1186/1750-1326-9-18

**Published:** 2014-05-19

**Authors:** Cassia R Overk, Anna Cartier, Gideon Shaked, Edward Rockenstein, Kiren Ubhi, Brian Spencer, Diana L Price, Christina Patrick, Paula Desplats, Eliezer Masliah

**Affiliations:** 1 Department of Neurosciences, University of California, San Diego, La Jolla, CA, USA; 2 Neuropore Therapies, Inc., San Diego, CA 92121, USA; 3 Department of Pathology, University of California, San Diego, La Jolla, CA, USA

**Keywords:** α-synuclein, Amyloid β oligomer, Dementia with Lewy body, Hippocampus, Human, mGluR5, Parkinsonism, Transgenic animal model

## Abstract

**Background:**

In dementia with Lewy bodies (DLB) abnormal interactions between α-synuclein (α-syn) and beta amyloid (Aβ) result in selective degeneration of neurons in the neocortex, limbic system and striatum. However, factors rendering these neurons selectively vulnerable have not been fully investigated. The metabotropic glutamate receptor 5 (mGluR5) has been shown to be up regulated in DLB and might play a role as a mediator of the neurotoxic effects of Aβ and α-syn in vulnerable neuronal populations. In this context, the main objective of the present study was to investigate the role of mGluR5 as a mediator of the neurotoxic effects of α-syn and Aβ in the hippocampus.

**Results:**

We generated double transgenic mice over-expressing amyloid precursor protein (APP) and α-syn under the mThy1 cassette and investigated the relationship between α-syn cleavage, Aβ, mGluR5 and neurodegeneration in the hippocampus. We found that compared to the single tg mice, the α-syn/APP tg mice displayed greater accumulation of α-syn and mGluR5 in the CA3 region of the hippocampus compared to the CA1 and other regions. This was accompanied by loss of CA3 (but not CA1) neurons in the single and α-syn/APP tg mice and greater loss of MAP 2 and synaptophysin in the CA3 in the α-syn/APP tg. mGluR5 gene transfer using a lentiviral vector into the hippocampus CA1 region resulted in greater α-syn accumulation and neurodegeneration in the single and α-syn/APP tg mice. In contrast, silencing mGluR5 with a lenti-shRNA protected neurons in the CA3 region of tg mice. *In vitro,* greater toxicity was observed in primary hippocampal neuronal cultures treated with Aβ oligomers and over-expressing α-syn; this effect was attenuated by down-regulating mGluR5 with an shRNA lentiviral vector. In α-syn-expressing neuronal cells lines, Aβ oligomers promoted increased intracellular calcium levels, calpain activation and α-syn cleavage resulting in caspase-3-dependent cell death. Treatment with pharmacological mGluR5 inhibitors such as 2-Methyl-6-(phenylethynyl)pyridine (MPEP) and 3-((2-Methyl-4-thiazolyl)ethynyl)pyridine (MTEP) attenuated the toxic effects of Aβ in α-syn-expressing neuronal cells.

The article "Hippocampal neuronal cells that accumulate α-synuclein fragments are more vulnerable to Aβ oligomer toxicity via mGluR5 – implications for dementia with Lewy bodies" was retracted in 2025. Reasons: duplicated images; overlap with earlier publications; unreliable data; concerns about the data.

**Conclusions:**

Together, these results support the possibility that vulnerability of hippocampal neurons to α-syn and Aβ might be mediated via mGluR5. Moreover, therapeutical interventions targeting mGluR5 might have a role in DLB.

## Background

Alzheimer’s disease (AD) and Parkinson’s disease (PD) are the leading causes of dementia and movement disorders in the aging population. It is estimated that over 5 million people live with these devastating neurological conditions in the US [1]. While in AD abnormal accumulation of misfolded amyloid-β protein (Aβ) in the neocortex and limbic system is responsible for the neurodegenerative pathology [2,3], in PD accumulation and propagation of α-synuclein (α-syn) has been centrally implicated in this condition [4-6]. The pathogenesis of AD and PD overlap in a heterogeneous group of conditions denominated jointly as Lewy body disease (LBD) [7,8], which includes dementia with Lewy bodies (DLB), Parkinson’s disease with dementia (PDD) and idiopathic PD (iPD). Direct and indirect interactions between α-syn and Aβ play a role in the pathogenesis of LBD [9-13]. Specifically, Aβ promotes the oligomerization and toxic conversion of α-syn [12,14]; Aβ worsens the deficits associated with α-syn accumulation [15,16]; Aβ and α-syn co-localize in membrane and caveolar fractions [13]; and Aβ stabilizes α-syn multimers that might form hetero-multimers in the membrane [13].

In DLB, neuronal populations degenerate in the neocortex, CA3 region of the hippocampus, and mid-spiny neurons in the striatum [17,18] Among the cell-autonomous factors that might render neurons vulnerable in DLB to the combined effects of Aβ and α-syn, it has been proposed that the expression profile of mGluRs might be a determinant for the degeneration of the hippocampal formation and neurons in DLB [19]. Considerable interest in mGluR5 [20] has developed in the last few years due to: **1)** its potential involvement in AD [21] and PD [22,23], **2)** the role of this receptor in learning and memory [24,25], **3)** mGluR5 is abundantly expressed in the neocortex, limbic system and caudoputamen [26]—brain regions selectively affected in AD and PD, and **4)** selective inhibitors of mGluR5, 2-methyl-6-(phenylethynyl)pyridine (MPEP) and 3-((2-Methyl-4-thiazolyl)ethynyl)pyridine (MTEP), are currently being considered as potential therapies for neurodegenerative disorders [23].

mGluR5 is more abundant in the hippocampal pyramidal neurons, the nucleus accumbens, and striatum of the basal ganglia and granular cells in the olfactory bulb (OB) [27,28], and is expressed at low levels in the cerebellum [26]. In AD and DLB the mGluR/phospholipase C (PLC) signaling pathways are impaired [29]. Moreover, Aβ dysregulates the PKC-dependent functions of mGluRs in cortical neurons [30] and the levels of mGluR5 are abnormal in AD patients, and are up regulated in the Down’s syndrome brains [31].

The article "Hippocampal neuronal cells that accumulate α-synuclein fragments are more vulnerable to Aβ oligomer toxicity via mGluR5 – implications for dementia with Lewy bodies" was retracted in 2025. Reasons: duplicated images; overlap with earlier publications; unreliable data; concerns about the data.

Remarkably, we have shown that in DLB and PD patients and α-syn transgenic (tg) mice there is increased expression of mGluR5 in the hippocampus and striatum [19]. In the 1-methyl-4-phenyl-1,2,3,6-tetrahydropyridine (MPTP) model of dopaminergic damage, activation of mGluR5 contributes to the neurodegenerative process [32] and mGluR5 blockers, such as MPEP, protect neurons from MPTP and 6-OH dopamine (DOPA) challenge [33-35].

Taken together, these studies suggest that mGluR5 might play a role as a mediator of the neurotoxic effects of Aβ and α-syn in AD and PD. In this context, the main objective of the present study was to investigate the role of mGluR5 as a mediator of the neurotoxic effects of α-syn and Aβ in the hippocampus. We found that degeneration of the CA3 region of the hippocampus in α-syn/APP double tg mice was associated with increased accumulation of α-syn and increased expression of mGluR5. Down regulation of mGluR5 was protective while ectopic overexpression of mGluR5 in the CA1 resulted in neurodegeneration. In α-syn expressing neuronal cells lines, Aβ oligomers promoted increased intracellular calcium levels, calpain activation and α-syn cleavage, resulting in caspase-3 dependent cell death. Together, these results support the possibility that vulnerability of hippocampal neurons to α-syn and Aβ might be mediated via mGluR5.

## Results

### Characterization and comparison of mRNA and protein expression in transgenic mouse lines expressing APP, α-syn and α-syn/APP

In order to understand the role of α-syn and Aβ in mediating neurodegeneration in the hippocampus via mGluR5, we generated α-syn/APP double tg mice by crossing mThy1-α-syn (Line 61) and mThy-1 APP (Line 41) (Figure 1A). We chose to cross these two specific tg lines to ensure co-expression of APP and α-syn in the same neuronal populations, at comparable levels, and because each individual line has shown robust pathology in vulnerable areas relevant to AD and PD [36,37]. Quantitative PCR (qPCR) analysis of mRNA isolated from brain tissue demonstrated the presence of comparable levels of hAPP mRNA in the APP and α-syn/APP tg mice (Figure 1B). Analysis of the same brain tissues for α-syn mRNA revealed comparable levels of hα-syn in both α-syn single tg and the α-syn/APP double tg mouse lines (Figure 1B). Double labeling and laser scanning confocal microscopy studies confirmed that in the α-syn/APP tg mice the same neuronal populations co-express human amyloid precursor protein (hAPP) and human α-syn (hα-syn) (Figure 1C). Consistent with the mRNA and immunohistochemical analysis, Western blot experiments also confirmed the presence of the native α-syn band at approximately 14 kDa in the non-tg and tg mice lines. In line with previous studies [9,12], the α-syn/APP tg mice displayed greater accumulation of α-syn (monomeric and oligomers) when compared to the α-syn tg mice (p-value < 0.05; Figure 1D and E). Western blot evaluation of APP revealed that full length (FL-) APP and Aβ levels were comparable between APP tg and α-syn/APP double tg mice (Figure 1F and G).

The article "Hippocampal neuronal cells that accumulate α-synuclein fragments are more vulnerable to Aβ oligomer toxicity via mGluR5 – implications for dementia with Lewy bodies" was retracted in 2025. Reasons: duplicated images; overlap with earlier publications; unreliable data; concerns about the data.

**Figure 1:** **Generation and characterization of tg mice expressing α-syn, APP or α-syn/APP under the mThy1 promoter. A**. Schematic representation of the α-syn and APP single tg mice. **B**. Levels of hAPP mRNA and hα-syn mRNA expressed as a ratio to the housekeeping gene GAPDH in non-tg APP, α-syn, and α-syn/APP tg mice. Mice express comparable levels of hAPP mRNA in the APP and α-syn/APP tg mice, as well as similar levels of α-syn mRNA in the α-syn and α-syn/APP tg mice. **C**. Laser scanning confocal microscopy studies confirmed that in the α-syn/APP tg mice the same neuronal populations co-express human amyloid precursor protein (hAPP) and human α-syn (hα-syn); scale bar = 10 μm. **D** Representative Western blot and **E** analysis showed the presence of native α-syn (14 kDa) in the membrane fraction all mice with the most enhanced accumulation of α-syn (monomeric and oligomers) occurring in α-syn/APP mice when compared to the α-syn tg mice (p-value < 0.05). **F**. Representative Western blot and **G** analysis of hAPP revealed that full length APP and Aβ levels were comparable between APP tg and α-syn/APP tg mice and APP. For analysis, N = 6 mice (3–4 months old) from each line were utilized. * = p-value < 0.05 by one-way ANOVA with a Tukey-Kramer *post hoc* analysis.

### Full-length α-syn and mGluR5 are increased in the CA3 pyramidal layer of the hippocampus in α-syn/APP mice compared to α-syn tg mice

To investigate the effects of the co-expression of α-syn and APP on mGluR5 levels in the hippocampus, immunocytochemical and image analysis was performed. We focused on the hippocampus because in previous studies we showed that the levels of mGluR5 were up regulated in the CA3 in a different single tg α-syn mouse line [19]. As expected, utilizing an antibody against total full-length α-syn that revealed the endogenous punctate pattern in the neuropil of the CA1 and CA3 regions in the non-tg and APP single tg mice (Figure 2A). In contrast, in the α-syn tg and α-syn/APP double tg mice α-syn was present in the neuronal cell bodies and had a significantly enhanced punctate pattern in the neuropil (Figure 2). In the CA3 there was a statistically significant increase in α-syn in the α-syn/APP double tg line compared with the α-syn single tg line (p-value < 0.05; Figure 2A and B); while in the CA1, the increase in α-syn in α-syn tg line was equivalent to the increase in the a-syn/APP double tg line, which were both significantly increased compared to non-tg mice (p-value < 0.05; Figure 2A and C).

The article "Hippocampal neuronal cells that accumulate α-synuclein fragments are more vulnerable to Aβ oligomer toxicity via mGluR5 – implications for dementia with Lewy bodies" was retracted in 2025. Reasons: duplicated images; overlap with earlier publications; unreliable data; concerns about the data.

**Figure 2:** **Comparison of the patterns of full-length α-synuclein in the hippocampus of APP, α-syn, and α-syn/APP tg mice.** Vibratome sections were immunostained with rabbit polyclonal antibody against full-length total α-syn (Millipore) **A**. Low- and high-magnification photomicrographs of the CA3 and CA1 regions of the hippocampus from non-tg, APP, α-syn, and α-syn/APP tg mice immunoreacted with anti-syn. Endogenous α-syn was observed in a punctate pattern in the neuropil of CA1 and CA3 in the non-tg and APP tg mice which was significantly enhanced in the α-syn and α-syn/APP tg mice. Moreover, α-syn and α-syn/APP tg mice also had α-syn in the neuronal cell bodies. **B**. Corrected optical densitometry analysis of the hippocampal CA3 region revealed that α-syn was significantly enhanced in both the α-syn and α-syn/APP tg mice compared to non-tg mice α-syn, and α-syn was significantly increased in the α-syn/APP double tg line compared with the α-syn single tg line. **C**. In the CA1, the increase in α-syn in α-syn tg line was equivalent to the increase in the α-syn/APP double tg line, which were both significantly increased compared to non-tg mice. Scale bars = 10 and 50 μm for the low and high magnifications, respectively. * = p-value < 0.05 by one-way ANOVA and Dunnett’s post hoc analysis compared to non-tg mice. # = p-value < 0.05 by one-way ANOVA and Tukey-Kramer post hoc analysis when, compared to α-syn/APP tg mice. For each analysis, N = 6 (3–4 months old) mice from each line were utilized.

Immunocytochemical analysis of mGluR5 revealed endogenous punctate pattern in the neuropil of non-tg mice in both the CA1 and CA3. As expected, in APP and α-syn single tg mice, mGluR5 was significantly increased in the cell bodies, as well as in the punctate pattern of the neuropil in the CA3 compared to non-tg mice (p-value < 0.05; Figure 3A and B). In α-syn/APP double tg mice, mGluR5 levels were statistically enhanced (p-value < 0.05) compared to α-syn single tg mice in the CA3, with mGluR5 increased in both the neuronal cell bodies, as well as in the neuropil (Figure 3A and B). While mGluR5 levels were increased in the CA3 across all tg lines, there was no increase in the CA1 compared to non-tg mice (Figure 3A and C), suggesting that the CA3 is selectively vulnerable to alterations in mGluR5 levels. Since there was an increased expression of mGluR5 in the CA3 pyramidal cell layer in α-syn/APP double tg mice, which paralleled the increase in FL-α-syn expression in the CA3 pyramidal cell layer of α-syn/APP mice compared to α-syn mice, sections were double-labeled for α-syn and mGluR5. Confocal microscopy of the CA3 pyramidal cell layer of the hippocampus confirmed that mGluR5 was increased in the presence of, and co-localized with, α-syn in both the α-syn tg and α-syn/APP double tg mouse lines compared to APP tg and non-tg mice (Figure 3D).

The article "Hippocampal neuronal cells that accumulate α-synuclein fragments are more vulnerable to Aβ oligomer toxicity via mGluR5 – implications for dementia with Lewy bodies" was retracted in 2025. Reasons: duplicated images; overlap with earlier publications; unreliable data; concerns about the data.

**Figure 3:** **Immunocytochemical analysis of mGluR5 in the hippocampus of APP, α-syn, and α-syn/APP tg mice.** Vibratome sections were immunostained with an antibody against mGluR5. **A**. Low- and high-magnification photomicrographs of the CA3 and CA1 regions of the hippocampus from non-tg, APP, α-syn, and α-syn/APP tg mice immunoreacted with anti-mGluR5. Endogenous mGluR5 was observed in a punctate pattern in the neuropil of CA1 and CA3 in the non-tg mice. In the CA3, but not the CA1 the APP, α-syn, and α-syn/APP tg mice had mGluR5 in the neuronal cell bodies, and the punctate staining in the neuropil was significantly enhanced. **B**. Corrected optical densitometry analysis of the hippocampal CA3 region revealed that mGluR5 was significantly enhanced across all tg mice compared to non-tg mice α-syn, and mGluR5 was significantly increased in the α-syn/APP double tg line compared with the α-syn single tg line. **C**. In the CA1, there was no significant difference in the amount of mGluR5 in any of the tg line compared to the non-tg line. **D**. Confocal imaging of CA3 hippocampus double-labeled with α-syn and mGLuR5 confirmed the presence and increase in mGluR5 with α-syn in both the α-syn and α-syn/APP tg mice. Scale bars = 10 and 50 μm for the low and high magnifications, respectively. * = p-value < 0.05 by one-way ANOVA and Dunnett’s post hoc analysis compared to non-tg mice. # = p-value < 0.05 by one-way ANOVA and Tukey-Kramer post hoc analysis when, compared to α-syn/APP tg mice. For each analysis, N = 6 (3–4 months old) mice from each line were utilized.

### Hippocampal CA3 but not CA1 pyramidal cells selectively vulnerable in APP, α-syn, and α-syn/APP tg mice

Based on the observation that mGluR5 and FL-α-syn are increased in the CA3 but not CA1, stereological analysis was performed to determine if the CA3 was selectively vulnerable to neurodegeneration in the APP, α-syn and α-syn/APP tg mouse lines (Figure 4). The number of NeuN-positive cells in the CA3 was significantly decreased by approximately 50% across all tg mouse lines (p-value < 0.05; Figure 4B) but remained unaffected in the CA1 pyramidal cell layer (Figure 4C). To further investigate the selective neurodegeneration in the hippocampal CA3 pyramidal layer, immunocytochemical analysis was performed with other markers including MAP 2 (dendritic marker), synaptophysin (pre-synaptic terminal marker), GFAP (astroglial cells), and Iba-1 (microglial cells). In the CA3 region of the non-tg mice, MAP 2-immunoreactivity (−ir) was found in the neuronal cell bodies and dendrites using confocal microscopy. In contrast, APP, α-syn and α-syn/APP tg mice displayed a reduction on MAP 2 immunolabeling in the CA3 region (p-value < 0.05; Figure 5A and B). The most dramatic loss in MAP 2-ir was in the α-syn/APP double tg mice, which showed a significant decrease in MAP 2-ir in the neuropil, both compared to non-tg mice (p-value < 0.01), as well as compared to α-syn single tg mice (p-value < 0.05; Figure 5A and B). Confocal microscopy and image analysis of synaptophysin in CA3 revealed abundant punctate staining in the pre-synaptic nerve terminals of non-tg mice (Figure 5A). While there was not much difference between in synaptophysin levels in non-tg and APP mice, the area of the neuropil that was synaptophysin-positive was significantly reduced in α-syn tg mice (p-value < 0.05) and even further reduced in the α-syn/APP tg mouse line (p-value < 0.01) in the CA3 of the hippocampus (Figure 5A and C).

The article "Hippocampal neuronal cells that accumulate α-synuclein fragments are more vulnerable to Aβ oligomer toxicity via mGluR5 – implications for dementia with Lewy bodies" was retracted in 2025. Reasons: duplicated images; overlap with earlier publications; unreliable data; concerns about the data.

**Figure 4:** **Decreased number of hippocampal CA3 but not CA1 pyramidal cells in APP, α-syn, and α-syn/APP tg mice. A**. Representative low- and high-photomicrographs of the hippocampal CA3 and CA1 regions of sections immunoreacted with NeuN. **B**. Stereological assessment of every 12^th^ section revealed a significant decrease in the number of neurons in the CA3. **C**. However, the number of neurons in the CA1 region was unaffected across all tg mouse line. Statistical analysis was conducted using one-way ANOVA post hoc Dunnett’s compared to non-tg mice; * p-value < 0.05. For analysis N = 3 (3–4 mos old) from each line were utilized.

**Figure 5:** **Hippocampal CA3 brain region selectively vulnerable in APP, α-syn, and α-syn/APP tg mice.** Immunocytochemical analysis was performed in the hippocampal CA3 pyramidal layer. **A**. Representative confocal, MAP 2- (dendritic marker) and synaptophysin- (pre-synaptic terminal marker), and photomicrographs of GFAP- (astroglial cells) and Iba-1- (microglial cells) ir. MAP 2-ir found in neuronal cell bodies and dendrites, was reduced in APP, α-syn and α-syn/APP tg mice. Synaptophysin was abundant in punctate staining in non-tg pre-synaptic nerve terminals and reduced in α-syn and α-syn/APP tg mice. GFAP-positive astroglial cells had small cell bodies with short processes in the non-tg mice, while APP, α-syn, and α-syn/APP tg mice had GFAP-positive astroglia with enlarged cell bodies and extended processes. Non-tg mice displayed strongly immunoreactive discrete Iba-1-immunoreactive microglia, which increased in APP, α-syn and α-syn/APP tg mice **B**. The percent area of MAP 2-ir neuropil was significantly decreased in all tg lines compared to non-tg mice, with the greatest loss in the α-syn/APP double tg mice. **C**. The percent of synaptophysin-ir neuropil area revealed a significant reduction in α-syn tg mice and further reduction in α-syn/APP tg mice. **D**. Optical density image analysis revealed a significant increase in GFAP-ir in the APP and α-syn tg mice, which was greatest in α-syn/APP double tg mice compared to non-tg mice. **E**. Image analysis confirmed a significant increase in the number of Iba-1-positive cells in APP and α-syn single tg mice, which was greatest in α-syn/APP double tg mice. * = p-value < 0.05 and ** = p-value < 0.01 by one-way ANOVA and Dunnett’s post hoc analysis compared to non-tg mice. # = p-value < 0.05 by one-way ANOVA and Tukey-Kramer post hoc analysis when compared to α-syn/APP tg mice. For each analysis, N = 6 (3–4 months old) mice from each line were utilized.

The article "Hippocampal neuronal cells that accumulate α-synuclein fragments are more vulnerable to Aβ oligomer toxicity via mGluR5 – implications for dementia with Lewy bodies" was retracted in 2025. Reasons: duplicated images; overlap with earlier publications; unreliable data; concerns about the data.

While the non-tg mice had GFAP-positive astroglial cells within small cell bodies and short processes, APP, α-syn, and α-syn/APP tg mice had GFAP-positive astroglia with enlarged cell bodies and extended processes (Figure 5A). Optical density image analysis revealed a significant increase in GFAP-ir in the APP (p-value < 0.05) and α-syn (p-value < 0.05), with the greatest increase in α-syn/APP double tg mice (p-value < 0.01) compared to non-tg mice in the CA3 region (Figure 5A and D). Non-tg mice displayed the presence of discrete Iba-1-immunoreactive microglia (Figure 5A). In the tg lines, morphological analysis revealed that APP, α-syn and α-syn/APP mice contained Iba-1-positive processes that were strongly Immunoreactive with increased staining of microglia processes. Image analysis confirmed a significant increase in the number of Iba-1-positive cells in APP (p-value < 0.05) and α-syn (p-value < 0.05) single tg mice, which was most increased in α-syn/APP double tg mice (p-value < 0.05) in the CA3 region (Figure 5E).

The article "Hippocampal neuronal cells that accumulate α-synuclein fragments are more vulnerable to Aβ oligomer toxicity via mGluR5 – implications for dementia with Lewy bodies" was retracted in 2025. Reasons: duplicated images; overlap with earlier publications; unreliable data; concerns about the data.

### Lentivirus mediated delivery of mGluR5 *in vivo* in the CA1 region is associated with increased vulnerability in a previously unaffected region

To investigate if increasing the levels of mGluR5 results in enhanced vulnerability of un-affected regions in the hippocampus, lentiviruses expressing either a control vector or mGluR5 was injected into the CA1 region of non-tg and tg mice (Figure 6A). As expected, following the injection of the lentivirus (LV) control, the levels and patterns of mGluR5 immunostaining in the CA1 where comparable among the non-tg and tg lines. Levels of α-syn were higher in the α-syn and α-syn/APP and comparable in the non-tg and APP tg mice (Figure 6B and C). Likewise the percent area covered by MAP 2 dendrites in the CA1 was similar among non-tg and tg lines (Figure 6B and C). In contrast, injection of the LV-mGluR5 resulted in a significant increase in mGluR5 in the neuronal cell bodies and dendrites in the CA1 of the hippocampus in the non-tg and tg lines (Figure 6D). There was a significant accumulation of α-syn in the CA1 region in the α-syn and α-syn/APP tg mice compared to non-tg and APP tg mice (Figure 6D and E). Moreover the accumulation of α-syn in the tg lines was greater in mice injected with LV-mGluR5 when compared to mice injected with the LV-control in the CA1 region. Confocal analysis of MAP 2 in the CA1 region showed that compared to the non-tg mice, APP and α-syn and α-syn/APP tg mice that were injected with LV-mGluR5 resulted in significant reduction of dendrites in the CA1 region (Figure 6D and E). Taken together, these results supports the possibility that increased expression of mGluR5 in the CA3 plays a role in the vulnerability of this region in tg mice and that ectopic over-expression of mGluR5 in the CA1 results in neurodegeneration.

**Figure 6:** **Creating mGLuR5-mediated vulnerability in the CA1 region via lentivirus delivery in vivo. A**. Schematic representation of lentivirus expressing either control vector or mGLuR5 that was injected unilaterally in the CA1 of the hippocampus. **B**. Representative photomicrographs and **C** image analysis of sections from mice injected with LV-control and immunoreacted with mGluR5, α-syn and MAP 2. Injecting LV-control had no effect on either non-tg or tg mice and was comparable to the initial characterization of these mice in which levels of mGLuR5 remained the same, α-syn increased in α-syn and α-syn/APP tg mice, and MAP 2-ir was unaffected. **D**. Representative photomicrographs and **E**. image analysis revealed that injection of the LV-mGluR5 resulted in a significant increase in mGluR5 in the neuronal cell bodies and dendrites in the CA1 of the hippocampus in the non-tg and tg lines. While α-syn remained unaffected by LV-mGluR5 with α-syn increased in α-syn and α-syn/APP tg mice, MAP 2-ir was significantly reduced in dendrites in the CA1 region. * = p-value < 0.05 and ** = p-value < 0.01 by one-way ANOVA and Dunnett’s post hoc analysis compared to non-tg mice. For each analysis, N = 6 (3–4 months old) mice from each line were utilized.

The article "Hippocampal neuronal cells that accumulate α-synuclein fragments are more vulnerable to Aβ oligomer toxicity via mGluR5 – implications for dementia with Lewy bodies" was retracted in 2025. Reasons: duplicated images; overlap with earlier publications; unreliable data; concerns about the data.

### Down-regulation of mGluR5 with a lentivirus sh-RNA protects hippocampal neuronal cells from the neurotoxic effects of Aβ and α-syn

Next we wanted to ascertain if down-regulating mGluR5 in the hippocampus would be protective in models of Aβ and α-syn toxicity. To investigate if reducing the levels of mGluR5 results in decreased toxicity in the hippocampus, lentiviruses expressing either a control vector or sh-mGluR5 was injected into the CA3 region of non-tg and tg mice (Figure 7A). In the LV-control group, the levels of mGluR5 were higher in the CA3 in the α-syn and α-syn/APP and comparable in the non-tg and APP tg mice (Figure 7B and C). The percent area covered by MAP 2 dendrites in the CA3 was significantly reduced in the APP, α-syn and α-syn/APP compared to non-tg and tg lines (Figure 7B and C). In contrast, injection of the LV-sh mGluR5 resulted in a significant decrease in mGluR5 in the neuronal cell bodies and dendrites in the CA3 of the hippocampus in the non-tg and tg lines (Figure 7D). There was a significant accumulation of α-syn in the CA3 region in the α-syn and α-syn/APP tg mice compared to non-tg and APP tg mice (Figure 7D and E). Confocal analysis of MAP 2 in the CA3 region showed that% area of the neuropil was comparable between the non-tg mice and the APP and α-syn and α-syn/APP tg (Figure 7D and E). Taken together, these results support the notion that reduced expression of mGluR5 in the CA3 is protective.

**Figure 7:** **Down-regulation of mGLuR5 in the CA3 region via shRNA lentivirus delivery is protective. A**. Schematic representation of lentivirus expressing either control vector or sh mGLuR5 that was injected unilaterally in the CA3 of the hippocampus. **B**. Representative photomicrographs and **C** image analysis of sections from mice injected with LV-control and immunoreacted with mGluR5, α-syn and MAP 2. Injecting LV-control had no effect on either non-tg or tg mice and was comparable to the initial characterization of these mice in which levels of mGLuR5, α-syn, and MAP 2-ir. **D**. Representative photomicrographs and **E**. image analysis revealed that injection of the LV-sh mGluR5 resulted in a significant reduction in mGluR5 in the neuronal cell bodies and dendrites in the CA3 of the hippocampus in the non-tg and tg lines. While α-syn remained unaffected by LV-sh mGluR5 with α-syn increased in α-syn and α-syn/APP tg mice, levels of MAP 2-ir were improved in the CA3 region. * = p-value < 0.05 and ** = p-value < 0.01 by one-way ANOVA and Dunnett’s post hoc analysis compared to non-tg mice. # = p-value < 0.05 by one-way ANOVA and Tukey-Kramer post hoc analysis when compared to α-syn/APP tg mice. For each analysis, N = 6 (3–4 months old) mice from each line were utilized.

The article "Hippocampal neuronal cells that accumulate α-synuclein fragments are more vulnerable to Aβ oligomer toxicity via mGluR5 – implications for dementia with Lewy bodies" was retracted in 2025. Reasons: duplicated images; overlap with earlier publications; unreliable data; concerns about the data.

To confirm the effects in an independent system *in vitro*, primary hippocampal neuronal cells were infected with an LV-sh-mGluR5 or LV-sh-Luc (control targeting luciferase) in combination with Aβ and α-syn. First we evaluated the expression of mGluR5; as expected, cells injected with LV-sh-Luc control expressed high levels of mGluR5 by immunocytochemistry (Figure 8A) and Western blot (Figure 8B). In contrast, cells infected with the LV-sh-mGluR5 displayed a significant 80% reduction in mGluR5 expression (Figure 8B). Next neuronal cells were co-infected with a LV-control or LV-α-syn and treated with vehicle or Aβ oligomers and analyzed by confocal microscopy for neuritic processes and α-syn levels (Figure 8C). Compared to the control, neuronal cells infected with LV-α-syn displayed 35-40% reduction in neurite length (Figure 8C and D), likewise neuronal cells infected with LV-control and challenged with Aβ oligomers alone resulted in 40-50% loss in neurite length that was worsened in cells infected with LV-α-syn (Figure 8C and D). Compared to control experiments using LV-sh-Luc, down modulation of mGluR5 with LV-sh-mGluR5 rescued the neuritic phenotype in both neuronal cells infected with LV-α-syn alone, treated with Aβ oligomers alone or in combination (Figure 8C and D). As expected neuronal cells infected with LV-α-syn expressed higher levels of α-syn (Figure 7C and E). Compared to vehicle treated cells, levels of α-syn where higher in infected cells treated with Aβ oligomers (Figure 8C and E). Down modulation of mGluR5 with LV-sh-mGluR5 had no effects on levels α-syn (Figure 8E). By LDH assay, compared to the control, neuronal cells infected with LV-control and challenged with Aβ oligomers alone resulted in greater neuronal cell death that was worsened in cells infected with LV-α-syn (Figure 8F). Compared to control experiments using LV-sh-Luc, down modulation of mGluR5 with LV-sh-mGluR5 protected neurons from the toxic effects of Aβ oligomers and -α-syn (Figure 8F).

**Figure 8:** **Blocking mGLuR5-mediated neuronal vulnerability to Aβ and α-syn in the hippocampal neurons via lentivirus shRNA delivery in vitro. A**. Confocal imaging and **B** Western blot of primary neuronal hippocampal cells, which endogenously express mGluR5. LV-sh-luciferase (control LV-sh) had no effect on the expression of mGluR5, while LV-sh-mGluR5 effectively reduced endogenous mGluR5 expression by 80%. **C**. Confocal microscopy of neuronal cells co-infected with LV-control or LV-α-syn in the presence of either LV-sh-Luc or LV-sh-mGluR5 and treated with vehicle or Aβ oligomers and double labeled with antibodies against α-syn and MAP 2. **D**. Image analysis revealed that neurite distance (MAP 2) was reduced 35-40% in neuronal cells infected with LV-α-syn, and when this system was challenged with Aβ oligomers, neurite length was further reduced to 40-50% of control. While LV-sh-Luc had no effect on neurite length in either the presence or absence of Aβ oligomers, down modulation of mGluR5 using LV-sh-mGluR5 rescued neurite length in neuronal cells treated with LV-α-syn, as well as with the combined toxicity of LV-α-syn and Aβ oligomers. **E**. Image analysis of α-syn revealed that neuronal cells infected with LV-α-syn expressed higher levels of α-syn compared to untreated cells, and that Aβ oligomers further increased this expression compared with cells only treated with LV-α-syn. Down modulation of mGluR5 with LV-sh-mGluR5 had no effect on α-syn levels. **F**. Neuronal survival by LDH, showing that down-modulation of mGluR5 is protective form the toxic effects of Aβ oligomers and α-syn. * = p-value < 0.05 by one-way ANOVA and Dunnett’s post hoc analysis compared to vehicle-treated uninfected neurons. # = p < 0.05 by one-way ANOVA and Tukey-Kramer post hoc analysis when compared to LV-α-syn + Aβ oligomers.

The article "Hippocampal neuronal cells that accumulate α-synuclein fragments are more vulnerable to Aβ oligomer toxicity via mGluR5 – implications for dementia with Lewy bodies" was retracted in 2025. Reasons: duplicated images; overlap with earlier publications; unreliable data; concerns about the data.

### Aβ and α-syn promotes cell death and abnormal calcium flux via mGluR5 in a neuronal cell line

Since previous have shown that mGluR5 might be involved in mediating the toxic effects of Aβ [30,38-42], and mGluR5 deficient mice or mice treated with mGluR5 inhibitors are protected from MPTP-induced toxicity in models of parkinsonism [25,34,43], we tested the role of mGluR5 in mediating toxicity in our system. For this purpose, the co-pathogenic mechanisms of Aβ and α-syn toxicity were investigated in the B103 rat neuroblastoma cells that were infected with LV-α-syn and treated with Aβ oligomers (10 μM) for 24 h. Levels of mGluR5 were analyzed, both by immunocytochemistry (Figure 9A and B) and WB (Figure 9C). The LV-control infected cells expressed low levels of mGluR5; in contrast, neuronal cells infected with LV-α-syn and challenged with control media or Aβ oligomers displayed an increase in mGluR5 levels over control (Figure 9C).

**Figure 9:** **α-Synuclein and Aβ effect mGluR5 to promote toxicity via increase intracellular calcium flux.** The co-pathogenic mechanisms of Aβ and α-syn toxicity were investigated in the B103 rat neuroblastoma cells infected with LV-α-syn and treated with Aβ oligomers. **A**. Immunocytochemistry, **B** image analysis and **C**. Western blot analysis of the levels of mGluR5 in B103 cells revealed the lowest levels in vehicle treated cells. mGluR5 was significantly increased in cells treated with Aβ or LV-α-syn alone; and mGluR5 levels were the highest in cells treated with both Aβ and LV-α-syn. Aβ increased levels of α-syn in cells where both were present. **D**. Intracellular calcium levels, as measured using the fluorescence-based FLIPR assay, revealed that Aβ treatment resulted in a two-fold increase in intracellular calcium compared to control cells. While LV-α-syn had no effect on its own, in combination with Aβ there was a three-fold increase in intracellular calcium, which was similar to the effect of treating cells with the mGluR5 agonist DHPG. Pretreating B103 cells with mGluR5 antagonists MPEP and MTEP prior to Aβ and LV-α-syn exposure attenuated the intracellular calcium increase. **E**. In the lactate dehydrogenase (LDH) toxicity assay, B103 cells were unaffected by LV-α-syn; however, the percent cell death dramatically increased when LV-α-syn was combined with Aβ oligomers. The mGluR5 agonist DHPG caused a similar level of cell death, while pretreatment with the mGluR5 antagonists MPEP and MTEP attenuated the neurotoxic effects and reduced cell death to levels similar to LV-α-syn alone. * = p-value < 0.05 by one-way ANOVA and Dunnett’s post hoc analysis compared to vehicle-treated control.

The article "Hippocampal neuronal cells that accumulate α-synuclein fragments are more vulnerable to Aβ oligomer toxicity via mGluR5 – implications for dementia with Lewy bodies" was retracted in 2025. Reasons: duplicated images; overlap with earlier publications; unreliable data; concerns about the data.

Since activation of mGluR5 results in increased intracellular calcium [20] and both α-syn [44] and Aβ [45,46] raise this ion, intracellular calcium was measured as previously described using fluorescence-based assay, FLIPR (Molecular Devices). In the LV-control infected cells, Aβ-treated cells displayed an approximate two-fold increase in intracellular calcium compared to control cells (Figure 9D). Treatment of LV-α-syn cells with the mGluR5 agonist- DHPG (1 μM, 24 h) showed similar results to the Aβ-treated group (Figure 9D). In the LV-α-syn infected cells, Aβ challenge resulted in approximate three-fold increase in intracellular calcium compared to control cells (Figure 9D). The combined effects of α-syn and Aβ on intracellular calcium levels were attenuated upon pre-treatment with the mGluR5 antagonists – MPEP (200 μM) and MTEP (20 μM) (Figure 9D). Using the lactate dehydrogenase (LDH) toxicity assay we found that while LV- α-syn infected cells displayed low toxicity, Aβ enhanced LV-α-syn toxicity to approximately three-times basal levels (p < 0.001) comparable to the toxicity levels of the mGluR5 agonist -DHPG (Figure 9E). The combined neurotoxic effects of LV-α-syn and Aβ were attenuated upon pre-treatment with the mGluR5 antagonists, MPEP and MTEP (Figure 9E). Together, these results support the possibility that α-syn and Aβ promote toxicity via increase intracellular calcium flux than in turn could activate proteases.

The article "Hippocampal neuronal cells that accumulate α-synuclein fragments are more vulnerable to Aβ oligomer toxicity via mGluR5 – implications for dementia with Lewy bodies" was retracted in 2025. Reasons: duplicated images; overlap with earlier publications; unreliable data; concerns about the data.

### Aβ promotes calpain mediated α-syn fragmentation and caspase-3 dependent cell death in α-syn-expressing neuronal cells

Since previous studies suggest that intracellular calcium results in calpain-I activation and C-terminus cleavage of α-syn (Figure 10A), LV-α-syn infected B103 neuronal cells were treated with Aβ and analyzed by WB. Remarkably, in cells treated with Aβ (10 μM, 24 h), the levels of FL-α-syn in the cytosolic fraction (soluble) were significantly increased (Figure 10B), while in the membrane fraction (insoluble) two immunoreactive bands were observed. An antibody specific for the C-terminal (CT) fragment of α-syn [47] confirmed that the shorter fragment generated was a CT-α-syn (Figure 10B). By confocal microscopy, LV-α-syn infected B103 cells treated with Aβ displayed increased CT-α-syn-ir (Figure 10C and D; p-value < 0.05). This suggests that proteolytic enzymes in the presence of Aβ might cleaved α-syn. Previous studies suggest that calpain-I (Figure 10A) might be involved in this process [48-51]. Consistent with this possibility, analysis of β-spectrin degradation by immunoblot showed that in LV-α-syn infected B103 cells treated with Aβ had an increased generation of β-spectrin fragments at 145/150 kDa and at 120 kDa (Figure 10E). FL β-spectrin is a 240 kDa protein, while a 145/150 kDa doublet is indicative of calpain cleavage, and the 120 kDa fragment is indicative of caspase-3 cleavage. The calpain-I mediated generation of CT α-syn in Aβ- treated cells was associated with activation of caspase-3 as reveled by immunocytochemical analysis (Figure 9F) and increased cell death by LDH (Figure 10G). Consistent with these findings, pre-treatment with calpain-I (calpeptin IV) or caspase-3 (z-DEVD-FMK) inhibitors significantly reduced cell death in LV-α-syn infected neuronal cells treated with Aβ (Figure 10G). Moreover, after 24 h incubation, co-IP analysis showed that α-syn interacts with caspase-3 (Figure 10H).

**Figure 10:** **Aβ promotes calpain mediated α-syn fragmentation and caspase-3 dependent cell death in α-syn-expressing neuronal cells. A**. Diagrammatic representation of calpain-mediated α-syn cleavage resulting in C-terminus truncation of α-syn. **B**. Representative Western blot showing increased levels in both FL-α-syn (14 kDa) in the cytosolic (single band) and membrane (double band) fractions, as wells as an increase in C-terminus cleavage of α-syn (12 kDa) when cells were pre-treated with Aβ. **C**. Representative confocal microscopy and **D** image analysis of B103 neuroblastoma cells treated with combinations of LV-α-syn and/or Aβ oligomers revealed increased CT-α-syn-ir (* p < 0.05; one-way ANOVA and Dunnett’s post hoc analysis compared to LV-α-syn treated with vehicle). **E**. Increased β-spectrin degradation by calpain and caspase-3, in the presence of LV-α-syn and Aβ. **F**. Caspase-3 activity was increased in cells treated with Aβ alone and combined with LV-α-syn. * p < 0.05; one-way ANOVA and Dunnett’s post hoc analysis compared to uninfected, vehicle-treated control. **G**. Calpain and caspase inhibitors rescued cell death induced by combined toxicity of Aβ and LV-α-syn. **H**. Co-ip of α-syn and caspase-3 in the presence of Aβ.

The article "Hippocampal neuronal cells that accumulate α-synuclein fragments are more vulnerable to Aβ oligomer toxicity via mGluR5 – implications for dementia with Lewy bodies" was retracted in 2025. Reasons: duplicated images; overlap with earlier publications; unreliable data; concerns about the data.

### Accumulation of CT α-syn and caspase-3 activation in α-syn/APP tg mice

To verify the effects on α-syn truncation in an *in vivo* model, Aβ and caspase-3 activation was determined using immunocytochemical and western blot analysis was performed. By confocal microscopy, APP and α-syn tg mice displayed a moderate increase in activated caspase-3-ir in the CA3 region of the hippocampus while the bigenic α-syn/APP mice showed an even greater increase compared to non-tg controls, (Figure 11A and B). Likewise, immunocytochemical analysis with an antibody against CT-α-syn showed a 0.5 to 1 fold increase in the single tg mice, while in the α-syn/APP tg mice displayed a 2.5 fold increase in the accumulation of CT- α-syn in the CA3 of the hippocampus (Figure 11C and D). By Western blot analysis using an antibody against CT- α-syn, detected a 12 kDa fragment at low levels in the single tg mice, while higher levels were detected in the α-syn/APP tg mice (Figure 11E and F). Moreover and consistent with the immunocytochemical analysis, levels of mGluR5 were higher in the α-syn and in the α-syn/APP tg mice compared to non-tg control mice (Figure 11E and F).

**Figure 11:** **Accumulation of CT α-syn and caspase-3 activation in α-syn/APP tg mice. A**. Confocal images and **B** image analysis of increased caspase-3 activation in the hippocampal CA3 region. While caspase-3 was significantly increased in all tg lines compared to non-tg mice, the most dramatic increase was in the α-syn/APP tg mice. **C**. Photomicrographs and **D** image analysis of C-terminal α-syn accumulation of α-syn CT fragments. Accumulation of CT-α-syn was significant in the α-syn tg line and was most significantly increased in the α-syn/APP tg line. **E**. Representative Western blot and **F**. immunoblot analysis showing increased levels of α-syn CTF and mGluR5 in APP, SYN, and SYN/APP tg mice. * = p-value < 0.05, and ** = p-value < 0.01 by one-way ANOVA and Dunnett’s post hoc analysis compared to non-tg mice. For each analysis, N = 6 (3–4 months old) mice from each line were utilized.

The article "Hippocampal neuronal cells that accumulate α-synuclein fragments are more vulnerable to Aβ oligomer toxicity via mGluR5 – implications for dementia with Lewy bodies" was retracted in 2025. Reasons: duplicated images; overlap with earlier publications; unreliable data; concerns about the data.

Taken together these results are in agreement with the in vitro experiments and suggest that vulnerability of hippocampal neurons to α-syn and Aβ might be mediated via mGluR5 via calpain and caspase-3 activation resulting in CT-truncation of α-syn.

## Discussion

The present study showed that in single tg as well as in α-syn/APP tg mice the vulnerability of the CA3 region of the hippocampus to the combined effects of α-syn and Aβ are associated with increased mGluR5 and CT-α-syn accumulation. Moreover, while mGluR5 gene transfer into the CA1 region (that otherwise was preserved) resulted in neurodegeneration, silencing mGluR5 in the CA3 was protective in the single and α-syn/APP tg mice. In agreement with the *in vivo* studies, Aβ toxicity was enhanced in α-syn expressing neuronal cell cultures and the effect was attenuated by down-regulating mGluR5 with an shRNA lentiviral vector or pharmacologically with MPEP/MTEP. In α-syn expressing neuronal cells, Aβ oligomers promoted increased intracellular calcium levels, calpain-I activation and α-syn cleavage resulting in caspase-3 dependent cell death.

These findings are consistent with our previous study showing that mGluR5 is elevated in the hippocampus of DLB patients, as well as in α-syn tg mice [19]. While in the previous study we analyzed PDGF-α-syn (line D) mice [19], for this new study we investigated the mThy1-α-syn (line 61), as well as crosses with the mThy1-APP mutant tg mouse model of DLB. This bigenic mThy1-α-syn/APP mutant tg line is new and has not been reported before. These lines were selected to ensure expression of α-syn and APP in the same neuronal populations and because the high levels of expression in the hippocampus and the extent of the α-syn and Aβ pathology [36,37]. Thus while for the previous study we focused on the effects of α-syn alone, for this study the emphasis was in investigating the combined effects of α-syn and Aβ and the downstream consequences on vulnerability and degeneration of hippocampal neurons. In the single and α-syn/APP tg mice neurodegeneration was only observed in CA3 but not in CA1. In contrast, injection of LV-mGluR5 resulted in degeneration of the CA1 region, while down-regulating mGluR5 in tg mice and in neuronal cultures was protective from the toxic effects of α-syn and Aβ. The mechanisms are not completely clear; however, one possibility is that α-syn aggregates might interfere with mGluR5 internalization via interactions with β-arrestin, which is involved in mGluR5 re-cycling [19]. Higher levels of mGluR5 in selected neuronal populations might render them more sensitive to the effects of excitatory agonists, such as glutamate and potentially Aβ.

The article "Hippocampal neuronal cells that accumulate α-synuclein fragments are more vulnerable to Aβ oligomer toxicity via mGluR5 – implications for dementia with Lewy bodies" was retracted in 2025. Reasons: duplicated images; overlap with earlier publications; unreliable data; concerns about the data.

The combined toxic effects of α-syn and Aβ via mGluR5 appeared to involve truncation of α-syn mediated by calpain-I. Previous studies have shown that c-terminally truncated α-syn is more prone to aggregate and to lead to neurotoxicity [52-55]. Both in the brains of patients with DLB/PD as well as in our α-syn tg mice [51] and in BAC-α-syn rats [56], c-terminally truncated α-syn is elevated. Among the proteases involved, calpain-I has been shown to play an important role [48]. The c-terminally truncated fragment we detected was consistent with calpain-I cleavage site as previously reported [51]. In our model, one possibility supported by the in vitro studies is that Aβ/α-syn interacts with mGluR5 might result in increased intracellular calcium that in turn could activate calpain-I triggering α-syn truncation and further aggregation. This is consistent with the known role of mGluR5 hyper-excitation mediated by Aβ [42,57].

The role of mGluR5 in AD and PD has been the subject of considerable interest because of the potential for a therapeutic target [58]. It has been shown that in AD the Aβ oligomers interact with mGluR5 [42,59] and that Aβ dysregulates astroglial mGluR5 and calcium signaling [60]. In addition, inhibition of mGluR5 is neuroprotective against Aβ toxicity [40] and mGluR5 is up regulated in Down syndrome [31]. In PD and related models, modulation of mGluR5 ameliorates the deficits in the MPTP treated mice [61] and 6-OH DOPA model [62].

Previous studies support the notion that α-syn and Aβ interact [63]. In Lewy body disease Aβ deposition is associated with α-syn lesions [9] and in crosses between PDGF-APP mutant and PDGF-α-syn, the α-syn pathology and related deficits are exacerbated [12]. Similar results have been reported when crossing 3xTg-AD mice with mPrP-α-syn A53T tg mice [15] and between PDGF-α-syn and mThy1-APP mutant tg mice [13]. In addition, α-syn mediated synapse damage is enhanced by Aβ [64] and α-syn and Aβ cross-seed [13,14,65,66].

## Conclusions

In order to understand the role of α-syn and Aβ in mediating neurodegeneration in the hippocampus via mGluR5, we generated α-syn/APP double tg mice by crossing mThy1-α-syn (Line 61) and mThy-1 APP (Line 41). In this model full-length α-syn and mGluR5 were increased in the CA3 pyramidal layer of the hippocampus in α-syn/APP mice compared to α-syn tg mice. This was the same region of the hippocampus that was selectively vulnerable in APP, α-syn, and α-syn/APP tg mice. Lentivirus-mediated delivery of mGluR5 *in vivo* in the CA1 region, which was previously unaffected in the tg mice lines, led to increased vulnerability. Down-regulating or pharmacologically blocking mGluR5 protected hippocampal neurons from the neurotoxic effects of Aβ and α-syn. Further experiments suggested that the vulnerability of hippocampal neurons to α-syn and Aβ might be due to calcium influx mediated through mGluR5 via calpain and caspase-3 activation resulting in CT-truncation of α-syn. Together, these results support the possibility that vulnerability of hippocampal neurons to α-syn and Aβ might be mediated via mGluR5. Moreover, therapeutical interventions targeting mGluR5 might have a role in DLB.

The article "Hippocampal neuronal cells that accumulate α-synuclein fragments are more vulnerable to Aβ oligomer toxicity via mGluR5 – implications for dementia with Lewy bodies" was retracted in 2025. Reasons: duplicated images; overlap with earlier publications; unreliable data; concerns about the data.

## Material and methods

### Generation of mThy-1 hAPP, hα-synuclein, and α-syn/APP transgenic mice

The University of California at San Diego’s animal subjects committee approved all experiments. Mice expressing human (h)α-syn-bearing under the neuronal mThy-1 promoter cassette (provided by Dr. H. van der Putten, Ciba-Geigy, Basel, Switzerland) were generated as previously described [37]. Mice expressing hAPP751 cDNA containing the London (V717I) and Swedish-(K670M/N671L) mutations under the regulatory control of the murine (m)Thy-1 gene (mThy1-hAPP751) were generated as previously described [36]. These single tg mice were then cross-bred to generated mThy-1 α-syn/APP double tg mice.

### Construction of lentiviral vectors

The mouse mGluR5 cDNA was cloned into the 3^rd^ generation lentivirus vector by PCR addition of the ApaI and BamHI restriction sites. This vector contains the human CMV promoter driving transgene expression and the WPRE element for increased mRNA stability. The sh-mGluR5 (GCA ACA TCC CGA ACA GT AA) was cloned into the pSI-H1-copGFP vector (SBI Vector) containing the H1 promoter. The control shRNA lentivector (LV-sh-Luc) contains an shRNA directed against firefly luciferase. Lentiviruses expressing -α-syn, mGluR5, sh-mGluR5, sh-luciferase or empty vector (as controls) was prepared by transient transfection in 293 T cells. The LV-α-syn has previously been characterized [67]. Lentivirus vectors were prepared by transient transfection of the 3 packaging plasmids and the vector plasmid in 293 T cells as previously described [68,69].

### Mouse lines and intracerebral injections of lentiviral vectors

A cohort of n = 48 (n = 24 LV-control and n = 24 LV-mGluR5) mice were divided into the following groups: a) non-tg, b) APP, c) α-syn and d) α-syn/APP tg mice (6 month old, n = 6 with LV-control and n = 6 LV-mGluR5 per group), were injected with 3 μL of the lentiviral preparations (2.5 × 10^7^ TU) into the hippocampus CA1 region (using a 5 μL Hamilton syringe). Similarly a cohort of n = 48 were injected with LV-control (n = 24) and LV-sh mGluR5 (n = 24). Briefly, as previously described [70], mice were placed under anesthesia on a Koft stereotaxic apparatus and coordinates (hippocampus: AP 2.0 mm, lateral 1.5 mm, depth 1.3 mm) were determined as per the Franklin and Paxinos atlas [71]. The lentiviral vectors were delivered using a Hamilton syringe connected to a hydraulic system to inject the solution at a rate of 1 μL every 2 min. To allow diffusion of the solution into the brain tissue, the needle was left for an additional 5 min after the completion of the injection. Mice survived for 3 months after the lentiviral injection.

The article "Hippocampal neuronal cells that accumulate α-synuclein fragments are more vulnerable to Aβ oligomer toxicity via mGluR5 – implications for dementia with Lewy bodies" was retracted in 2025. Reasons: duplicated images; overlap with earlier publications; unreliable data; concerns about the data.

### Tissue preparation

Following NIH guidelines for the humane treatment of animals, mice were anesthetized with chloral hydrate and flush-perfused transcardially with 0.9% saline. Brains were removed and divided in sagittal sections. The right hemi-brain was post-fixed in phosphate-buffered 4% PFA (pH7.4) at 4°C for 48 h for neuropathological analysis, while the left hemibrain was snap-frozen and stored at −70°C for subsequent RNA and protein analysis.

### RNA extraction and quantification of mRNA by real time-PCR analysis

RNA was extracted from mice in triplicate using the RNAeasy kit (QIAGEN, Germantown, MD, USA) [37], and quantified by spectrophotometer readings. For cDNA synthesis, 1 μg total RNA was reverse transcribed using iScript cDNA Synthesis kit (BioRad, Hercules, CA, USA). Real Time-PCR (RT-PCR) experiments were performed using the iQ5 Detection System (BioRad, Hercules, CA, USA). Amplification was performed on cDNA equivalent to 25 ng total RNA with 1 × iQ SYBRGreen Supermix (BioRad, Hercules, CA, USA). Template PCR reactions were performed in triplicate and run in duplicate using the following PCR cycling parameters: 50°C for 2 min, 95°C for 10 min, and 40 cycles of 94°C for 15 s, 60°C for 1 min followed by a dissociation protocol to verify the presence of a single product for each amplicon. The amount of cDNA was calculated by the comparative threshold cycle method and expressed using mouse actin as an internal control.

### Immunohistochemical analysis

Analysis was performed using free-floating, 40 μm thick, vibratome cut, blind-coded sections, as previously described [51,72]. Briefly, sections were incubated overnight at 4°C with antibodies against total α-syn (1:500, affinity purified rabbit polyclonal, Millipore) [73], C-terminus α-syn (SYN105, mouse monoclonal) [51], and mGluR5 (1:500; Millipore), followed by biotin-tagged anti-rabbit or anti-mouse IgG1 (1:100, Vector Laboratories, Inc., Burlingame, CA) secondary antibodies, Avidin D-HRP (1:200, ABC Elite, Vector), and visualized with diaminobenzidine (DAB). Background levels were obtained in tissue sections immunostained in the absence of primary antibody. Therefore: corrected optical density = optical density – background. Sections were scanned with a digital Olympus bright field digital microscope (BX41).

The article "Hippocampal neuronal cells that accumulate α-synuclein fragments are more vulnerable to Aβ oligomer toxicity via mGluR5 – implications for dementia with Lewy bodies" was retracted in 2025. Reasons: duplicated images; overlap with earlier publications; unreliable data; concerns about the data.

Analysis of neurodegenerative pathology was performed in vibratome sections immunolabeled with antibodies against the dendritic marker microtubule-associated protein-2 (MAP 2; 1:500, Millipore), pan-neuronal marker NeuN (1:500, Millipore), astroglial marker glial fibrillary acidic protein (GFAP, 1:1000, Millipore) the microglial cell marker Iba-1 (Wako Laboratories, mouse monoclonal), activated caspase-3 (1:500; Cell Signaling) and synaptic marker synaptophysin (SY38, 1:500, Millipore) [51,73]. Sections reacted with antibodies against NeuN (1:4,000; Millipore), GFAP and Iba-1 were incubated with biotinylated secondary antibodies, Avidin D-HRP, and visualized with DAB. Sections reacted with antibodies against MAP 2 and synaptophysin were visualized with FITC-tagged secondary antibody or the Tyramide Signal Amplification™ Direct (Red) system (1:100, NEN Life Sciences, Boston, MA), respectively, mounted under glass coverslips with anti-fading media (Vector Laboratories), and imaged with the laser scanning confocal microscope (LSCM) (MRC1024, BioRad).

### Image analysis and stereology

Sections immunostained with antibodies against α-syn, mGluR5 and GFAP were analyzed with a digital Olympus bright field digital microscope (BX41). For each case a total of three sections (4 digital images per section at 400 × magnification) were obtained from the CA1 and CA3 region of the hippocampus and analyzed as previously described with the image J program (NIH) to obtain optical density, levels were corrected to background. Sections labeled with Iba-1, were analyzed utilizing the Image-Pro Plus program (Media Cybernetics, Silver Spring, MD) (10 digital images per section at 400 × magnification) and analyzed in order to estimate the average number of immuno-labeled cells per unit area (mm2) and the average intensity of the immunostaining (corrected optical density).

The numbers of NeuN-immunoreactive neurons were estimated utilizing unbiased stereological methods [74]. Hemisected brains were cut as serial sections and every 12th section containing the neocortex, hippocampus and striatum was outlined using an Olympus BX51 microscope running StereoInvestigator 8.21.1 software (Micro-BrightField, Cochester, VT). Grid sizes for the hippocampal CA3 and CA1 pyramidal layers were: 150 × 150 and 300 × 300 μm, respectively and the counting frames were 30 × 30 and 50 × 50 μm, respectively. Perikarya within section approximately 480 μm apart were counted only if the first recognizable profile came into focus within the counting frame. A systematic sampling of the regions of interests was made from a random starting point. Full penetration of the section by the antibody was confirmed by focusing throughout the entire Z-axis. The average coefficient of error for each region was 0.09. Sections were analyzed using a 100 × 1.4 PlanApo oil-immersion objective. The average mounted tissue thickness was 10.1 μm, and a 5 μm high disector allowed for 2 μm top and bottom guard-zones.

The article "Hippocampal neuronal cells that accumulate α-synuclein fragments are more vulnerable to Aβ oligomer toxicity via mGluR5 – implications for dementia with Lewy bodies" was retracted in 2025. Reasons: duplicated images; overlap with earlier publications; unreliable data; concerns about the data.

Sections immunolabeled with antibodies against MAP 2 and synaptophysin were serially imaged with the LSCM (MRC1024, BioRad) and analyzed with the Image J program (NIH), as previously described [75]. For each mouse, a total of 3 sections were analyzed and for each section, 4 fields in the CA1 and CA3 of the hippocampus were examined. Results were expressed as percent area of the neuropil occupied.

### Double immunolabeling and fluorescence co-labeling

To determine the co-localization between α-syn and APP, as well as mGluR5 and cleaved caspase-3, double-labeling experiments were performed as previously [75]. Sections were immunolabeled with the following pairs of antibodies: a) human α-syn (SYN211, mouse monoclonal, Millipore) and APP (6E10, mouse monoclonal Covance), b) human α-syn (SYN211, mouse monoclonal, Millipore) and mGluR5 (Millipore, rabbit polyclonal) and c) cleaved caspase-3 (Cell Signaling, rabbit polyclonal) and C-terminal α-syn (SYN105 mouse monoclonal). All sections were processed simultaneously, and experiments were performed in triplicate. The FL and CT α-syn was detected with the Tyramide Red (NEN Life Sciences) whereas APP and mGluR5 were detected with FITC-tagged antibodies (1:75, Vector, Burlingame, CA). Sections were imaged with a Zeiss 63X1.4 objective on an Axiovert 35 microscope (Zeiss) with an attached MRC1024 laser scanning confocal microscope (LSCM) system (BioRad) [75].

### Immunoblot analysis in co-immunoprecipitation

The levels of α-syn, APP and mGluR5 in mouse brains, as well as the levels of α-syn, mGluR5, brain spectrin and CT-α-syn in neuronal cultures were analyzed using lysate that were extracted and fractioned into soluble and insoluble fractions by ultracentrifugation [75]. Protein (20 μg/lane) was loaded onto 4-12% SDS/PAGE gels and blotted onto PVDF membranes, incubated with specific antibodies, followed by HRP-tagged secondary antibodies (1:5,000; Santa Cruz Biotechnology). Bands were visualized by enhanced chemiluminescence (ECL, PerkinElmer, Boston, MA) and analyzed with a quantitative Versadoc XL imaging apparatus (BioRad). β-Actin (1:3,000) was the loading control.

The article "Hippocampal neuronal cells that accumulate α-synuclein fragments are more vulnerable to Aβ oligomer toxicity via mGluR5 – implications for dementia with Lewy bodies" was retracted in 2025. Reasons: duplicated images; overlap with earlier publications; unreliable data; concerns about the data.

To detect interactions between α-syn and caspase-3 co-immunoprecipitation was performed as previously described [76] in neuronal cell lines infected with LV-α-syn and treated with Aβ oligomers. Briefly, immunoprecipitation assays were carried out essentially as previously described [77]. The lysates were then centrifuged for 20 min at 12,000 rpm, and the protein concentrations were determined with a BCA protein assay kit. Three hundred μg of each of the supernatants was incubated with 1 μg of the antibody against α-syn, overnight at 4°C. Then the immunocomplexes were adsorbed to protein A-Sepharose 4B or protein G-Sepharose (Amersham, Piscataway, NJ). After extensive washing with immunoprecipitation buffer, which contained 1% Trion X-100, samples were heated in NuPAGE SDS sample buffer (Invitrogen) for five min and subjected to gel electrophoresis on tris-tricine gels followed by immunoblot analysis with an antibody against caspase-3. The inverse immunoprecipitation with caspase-3 and immunoblotting with α-syn was also performed.

### Primary neuronal cultures treatments, lentiviral vectors and analysis

Hippocampal neuron cultures were prepared from P1 mouse hippocampi. Briefly, mouse hippocampi were dissected in HBSS dissecting media containing 4 mM NaHCO_3_ (7.5%) and 10 mM HEPES buffer. Neurons were then dissociated by enzymatic treatment with 0.25% trypsin in dissecting media for 15 min at 37°C, and subsequent mechanical disruption. Neurons were plated at medium density (45,000 cells/cm^2^) on poly-L-lysine coated coverslips (12 mm in diameter) in MEM plating media containing 1 mM sodium pyruvate, 0.6% glucose, 10% horse serum, and 2 mM glutamine. Cultures were placed in an incubator at 37°C under a humidified atmosphere of 5% CO_2_ in air for 2 hrs. The plating culture medium was then replaced and cultures were maintained in B27 supplemented Neurobasal media (Invitrogen) until 12 days *in vitro* (DIV). Primary neuronal cultures were infected with LV-control or LV-α-syn and with LV-sh-Luc or LV-mGluR5 after 48 hrs were treated with Aβ oligomers as previously described [76]. Natural Aβ was prepared according to Walsh et al. [78] (kindly provided by Dr. Eddie Koo) by incubating control CHO cells or CHO cells expressing APP V717F mutation (also referred as 7PA2 cells) with B27 conditioned media for 16 hrs. Total AΒ concentration was determined as previously described [79]. Neurons were treated with 80 pM of natural Aβ for 24 hrs. Hippocampal neurons were plated on coverslips were rinsed briefly in PBS and fixed with 4% paraformaldehyde (PFA) and 4% sucrose in PBS-MC (phosphate buffered saline with 1 mM MgCl_2_ and 0.1 CaCl_2_) for 10 min at room temperature. Neurons were then double immunolabeled as described above with antibodies against MAP 2 (Millipore) and α-syn (SYN211, Millipore). α-Syn was detected with the Tyramide Red (NEN Life Sciences) whereas MAP 2 was detected with FITC-tagged antibodies (1:75, Vector, Burlingame, CA). Coverslips were imaged with a Zeiss 63 × 1.4 objective on an Axiovert 35 microscope (Zeiss) with an attached MRC1024 laser scanning confocal microscope (LSCM) system (BioRad) [75] and analyzed with Image J to determine neurite length and levels of α-syn-ir (pixel intensity). The capacity of the LV-sh-mGluR5 at down-regulating mGluR5 was verified in coverslips by immunocytochemistry with an antibody against mGluR5 detected with Tryramide Red and by immunoblot as described above.

The article "Hippocampal neuronal cells that accumulate α-synuclein fragments are more vulnerable to Aβ oligomer toxicity via mGluR5 – implications for dementia with Lewy bodies" was retracted in 2025. Reasons: duplicated images; overlap with earlier publications; unreliable data; concerns about the data.

### Neuronal cell lines treatments, lentiviral vectors and analysis

The rat neuroblastoma cell line B103 was used for in vitro experiments because this cell line display neuronal features and we have shown that pathological features of synucleonopathies emerge when infected with LV-α-syn [69]. B103 cells were plated at 3.5×10^4^ cells/well on coverslips. After 6 hours cells were infected with LV-control, LV-α-syn (MOI = 50) and treated overnight later with Aβ oligomers (1 nM). Cells were then fixed in 4% paraformaldehyde and analyzed by immunocytochemistry for the expression of α-syn (Millipore), CT-α-syn (SYN105), caspase-3 (cell signaling) and mGluR5 (rabbit polyclonal) as described above. Cell lysates were divided by ultracentrifugation into soluble and insoluble fractions and analyzed by immunoblot for mGluR5, CT α-syn, α-syn and brain spectrin (Millipore) as described above.

To determine the involvement of mGluR5 in cytotoxicity, prior to the addition of Aβ oligomers, sets of cells infected with LV-control and LV-α-syn were pre-treated for 6 hrs with the mGluR5 antagonists MPEP hydrochloride (50 μM) (Tocris) and MTEP (50 μM) (Millipore) or the mGluR5 agonist DHPG Dihydroxyphenylglycine (10 μM) (Tocris) and analyzed for calcium levels and cytotoxicity. Cytotoxicity was assessed using the lactate dehydrogenase (LDH, CytoTox 96 assay, Promega) and MTT (3-(4,5-Dimethylthiazol-2-yl)-2,5-diphenyltetrazolium bromide, Roche) cell viability assays, as per manufacturer’s instructions, to measure levels of cell death. Assessment of calcium influx was carried out as previously described [13] using a modified protocol of the FLIPR 4 calcium assay (Molecular Devices, Sunnyvale, CA). Briefly, B103 cells were infected with lentiviral constructs. Cells were infected at a MOI of 30, and two days after infection, cells were plated at a density of 30,000 cells/well on Costar 96 well-black plates with flat clear bottom (Corning). After an additional 24 hrs of incubation, media was replaced by 100 μL of HBSS buffer, and 100 μL of calcium dye (FLUO-4 NW, Invitrogen) was added to each well. Cells were kept in the incubator at 37°C for 30 mins, followed by incubation in the dark at room temperature for an additional 30 mins before measuring fluorescence with an excitation/emission filter at 470-495/515-575 nm on a DTX 880 Multimode Detector (Beckman Coulter). As a positive control of calcium influx, 0.6 μg of ionomycin (Sigma, St. Louis, MO), was added to control wells.

The article "Hippocampal neuronal cells that accumulate α-synuclein fragments are more vulnerable to Aβ oligomer toxicity via mGluR5 – implications for dementia with Lewy bodies" was retracted in 2025. Reasons: duplicated images; overlap with earlier publications; unreliable data; concerns about the data.

Finally to ascertain the role of calpain-I and caspase-3 in neurotoxicity prior to the addition of Aβ oligomers, were pre-treated for 6 hrs with the calpain-I inhibitor calpastatin (50 nM) (Takeda) and the caspase-3 inhibitor N-Acetyl-Glu-Ser-Met-Asp-al (1 μM) (Sigma) followed by analysis of cytotoxicity by LDH as described above.

### Statistical analysis

All analyses used GraphPad Prism (version 5.0). Differences among means were assessed by one-way ANOVA with Dunnett’s post-hoc test when compared to non-tg and by Tukey-Kramer when comparing tg groups. Two-way ANOVA with repeated measures followed by a Bonferroni multiple comparisons post-hoc test was used for analyzing the interactions between groups and time. The null hypothesis was rejected at the 0.05 level.

## Competing interests

The authors declare that they have no competing interests.

## Authors’ contributions

CRO conceived and carried out the stereological studies and drafted the manuscript. AC performed in vitro studies with primary neuronal cell cultures. GS performed in vitro studies using neuroblastoma cell line. ER generated the tg mice and crosses. KU performed the initial characterization of the crosses. BS conceived/developed and performed experiments with mGluR5 and α-syn lentiviruses. DP conceived the role of mGLuR5 in DLB and contributed to in vitro characterization of mGLuR5 levels. CP performed and analyzed the immunoassays and the in vivo analysis. PD designed and performed the in vitro calcium studies. EM conceived the idea, contributed to the writing, and performed confocal microscopy analysis. All authors read and approved the final manuscript.
